# Construction of a Landscape Design and Greenery Maintenance Scheduling System Based on Multimodal Intelligent Computing and Deep Neural Networks

**DOI:** 10.1155/2022/8307398

**Published:** 2022-06-26

**Authors:** Mingfei Ji, Jianrong Lu, Xiaowei Zhang

**Affiliations:** ^1^Collaborative Innovation Center of Water Security for Water Source Region of Mid-Route Project of South-North Water Diversion of Henan Province, Nanyang Normal University, Nanyang 473061, China; ^2^College of Water Resource and Environment Engineering, Nanyang Normal University, Nanyang 473061, China; ^3^College of Forestry, Gansu Agricultural University, Lanzhou 730070, China

## Abstract

Digitalization brings challenges and new opportunities to the development of landscape gardening, “smart gardening,” which is a product of landscape gardening in response to the development of the digital era. Based on the multimodal intelligent computing method and deep neural network machine learning algorithm, this paper adopts “digital landscape design logic” to analyze and research smart gardens and digital design. The digital landscape design process and methods are discussed based on design logic, design basis, environment analysis, and results presentation, and the greenery maintenance scheduling system is constructed. The paper focuses on the digital implementation of the environmental analysis of the site and uses Rhino software and Grasshopper visual programming language to build parametric logic, establish parametric analysis models, and conduct a comprehensive analysis of the current environment. The main theme of the whole paper is a logical approach to digital landscape design for smart gardens, using digital technology tools from the perspective of smart garden thinking, combining quantitative analysis and qualitative design, and intervening in digital landscape garden planning and design to explore the application of digital technology and tools.

## 1. Introduction

With the development of the times, urban construction is changing day by day, the level of computer technology is advancing by leaps and bounds, and the progress of technology has also driven the development of various fields. The construction of ecological civilization should be in line with the development of the times, the basis for the realization of people's growing material needs and aspirations for a better life is an excellent living environment, and a beautiful and livable living environment in a modern society with rapid technological development requires the assistance of science and technology [1]. Smart gardens are the product of the development of smart cities and a means to promote the construction of urban life infrastructure, and the development model of smart cities promotes the transformation of the development model of smart gardens. Due to the development and application of big data, network technology, and 3S technology, the design mode of traditional gardens gradually changes towards the direction of smart gardens. In recent years, the construction of smart gardens and digitalization has now been commonly carried out in various industries. The rapid growth of digitization has brought many challenges to urban development. In the face of the increasingly complex elements and work of urban gardens, the traditional garden design method, which mainly relies on the designer's knowledge and experience, and aesthetic ability, this method has been difficult to meet the requirements of urban spatial planning due to the rapid development of cities and high standards and scientific, modern urban construction is in urgent need of vitality and innovation, keeping pace with the times, integrating science and technology into disciplinary research, building a perfect wisdom garden design method, and improving. We design an MOA algorithm, which is a multituple collaborative optimization algorithm, and the algorithm is designed with the multituple property in mind, which can be equated to the multituple property of the small habitat algorithm. In the algorithm, each queue node and its corresponding stack constitute a search group, as opposed to all search elements in the entire structure table, which represent the entire search tuple. During the search process, each search group maintains its independence, and global information is exchanged only when the queue nodes are sorted. The level of information, wisdom, refinement, science, and humanization of gardens should become the focus of the thinking of landscape gardeners at this stage [2].

As the development scale of landscape design continues to grow and respond to changes in the market environment, the business model also continues to change, leading to the evolution of the requirements for information management from local to overall, from headquarters to grassroots, and from simple to composite, and the construction of greenery maintenance scheduling also requires step-by-step optimization, upgrading, expansion, promotion, and transformation, which indicates that the demand for enterprise information management is from narrow to wide, from shallow to deep, and from simple to complex. Landscape design emphasizes art but not science, and qualitative design is much greater than quantitative analysis [3]. Due to technical limitations and the lack of platforms for communication with other disciplines, quantitative analysis lacks scientific guidance and is difficult or ineffective to carry out, making the current landscape design still largely dependent on the experience of designers, with the rationality and scientificity of the scheme to be proven and the assessment and prediction of the land suitability and ecological sustainability of the landscape lacking.

The main research content of this paper is to think from the perspective of wisdom gardening, using multimodal intelligent computing methods in the preplanning and design stage of wisdom gardening, through deep neural network algorithms, following digital design logic and design process, with the help of digital software and technological equipment, to make the landscape design and greenery maintenance scheduling more rational, wisdom, and refinement, where “wisdom” in this paper has two meanings: One is the wisdom in landscape design, through wise design means to achieve a humane, ecologically sustainable, harmonious state of man and nature. The second is the wisdom of science and technology, using modern technological means, such as digital dynamic models, VR technology, intelligent platforms, mobile Internet, intelligent monitoring systems, and other modern sciences and technologies to open the window of communication between man and nature.

Literature [4] argues that intelligent gardens should apply digital technology from the design stage, and the digital design approach and intelligent display of results can better promote intelligent construction and management at a later stage. Nowadays, the construction industry has started to implement digital design and construction, introduce BIM technology, and intervene in the whole process of construction to achieve the initial intelligence. Until now, the study of smart landscape design has also followed the trend of introducing GIS, BIM, and LIM technologies to digitally intervene in the construction of smart gardens. Literature [5] emphasizes that the application of BIM technology will improve the efficiency of various aspects of project planning, design, analysis, and evaluation, optimize the project design process, and transform the design logic; BIM technology was applied in the design process of smart gardens, where BIM technology simulates spatial entities through 3D virtual models and uses dynamic models of environmental space in the analysis and evaluation, planning, and design aspects to deepen designers' understanding of the project, deepen the analysis and excavation of project advantages and highlights, and improve design efficiency and project quality. In literature [6], remote sensing, GPS, monitors, sensors, and mobile smart terminals such as cell phones are used in the development of the technical framework of the landscape management system, and these smart devices can be used to view the current situation of the city, changes in the distribution of green areas, landscape maintenance, and management in real time and obtain the corresponding business data. Literature [7] collated the contents of current smart garden applications based on GIS technology, established comprehensive information management and monitoring platform, developed various smartboards of smart gardens, and realized, through GIS technology, the monitoring of landscape tourism sites, monitoring of classical gardens, information control of landscaping projects, video monitoring, map query of the location of attractions, and statistical analysis of data of different attractions. Xu [8] elaborated on the direction of smart garden applications, using sensors to monitor in real time the various environmental elements in the garden, such as temperature and humidity, CO_2_ concentration, uploading the detected information in the form of data to the background for data analysis, making intelligent irrigation, making early warning reports on pests and diseases based on the analysis results, and conducting information dissemination at the terminal and online reading and communication at the user end through the big data platform. For example, the public can conduct virtual tours of attractions, greening protection reports, and expert guidance and consultation online. In this way, the information, visualization, intelligence, and refinement of garden services and management are realized. In literature [9], an “intelligent garden” was created to conduct scientific planting and maintenance experiments. The designers developed a “visualization system” and a “virtual plant” to collect environmental data through environmental sensors, such as temperature, humidity, light intensity, soil moisture, conductivity, and pH, and then, based on these data, constructed a virtual environment in time and space axes. Models are constructed on temporal and spatial axes and these models are used to develop garden watering and fertilization schedules, plant growth condition monitoring, and growth prediction. The ultimate design goal of the “smart garden system” developed in literature [10] is to design a garden system that can obtain water in real time. The smartphone can be used to obtain temperature and weather information, take watering measures, and execute them through an application in the smartphone, where the virtual reality technology and the “intelligent decision-making system” are of reference value for the study of smart gardens. In literature [11], the main current digital design methods are sorted out and a preliminary and relatively accurate spectrum of the concept of digital planning and design of landscape gardens is delineated: one is the spectrum of computer-aided design, the second is the spectrum of digital design media and information management, and the third is the digital information model of landscape gardens. Corbaci et al. [12] summarized the core scientific issues facing the landscape gardening field at this stage as the synergy of ecology and form, the satisfaction of people's needs, and the innovation of design and practice. It is proposed that the integration of “interdisciplinary and cross-disciplinary” technologies and methods and the collaboration of “whole process and precise” design practices will be the future development and application trends of digital landscape technology in China's landscape gardening field. In literature [13], a general framework system for urban parks was constructed, and digital city-related technologies were analyzed in terms of data acquisition, storage, and sharing, and the application of digital systems was elaborated in terms of monitoring systems and web portals for security supervision systems. Carmona-Ribeiro and Carboni [14] used the artificial neural network BP algorithm model to establish ecological planning of urban landscape, and variables such as diversity, number of subdimensions, and aggregation of forest landscape patterns were input into the artificial neural network model and applied to the simulation and analysis planning of forest landscape pattern. Sas-Bojarska and Rembeza [15] learned the plan layout of real residential design schemes by Bayesian neural network algorithm, converted the plan layout into bubble diagrams using artificial supervised learning for artificial intelligence algorithm programs to count probabilities, and outputted the machine-learned design schemes with the help of connection tree and Castro tree algorithm.

In this paper, we will introduce a multimodal intelligent optimization algorithm and deep neural network algorithm to study the scheduling of gardening maintenance. Based on the existing research results, we will complete the design of the plant information function, climate information function, task information function, personnel information function, and scheduling management function based on system requirement analysis, using a multimodal intelligent optimization algorithm and deep neural network algorithm to complete the scheduling optimization design. Finally, the system functions and performance are tested. When designing this landscape maintenance scheduling management system, a long-term requirement needs to be designed to facilitate the system's functional services to be continuously increased in the subsequent process to meet the needs brought about by the development of the garden. The design of the system can not only improve the level of garden plant maintenance but also help to better carry out the daily maintenance of garden plants and can provide useful information to the daily management of garden plants in a timely and accurate manner, to better serve the management of garden plants and prevent the phenomenon of blindness, which is conducive to the improvement of social, ecological, and economic benefits.

## 2. A Study of Multimodal Intelligent Computing and Deep Neural Network Approach in Landscape Design and Greenery Maintenance Scheduling

### 2.1. Multimodal Intelligent Computing and Deep Neural Network Algorithm Selection

Multimodal machine learning aims to use machine learning methods to achieve the ability to process and understand multisource modal information. Currently, multimodal machine learning can be divided into five main research directions: multimodal representation learning, modal transformation, modal alignment, multimodal information fusion, and multimodal cooperative learning. While unimodal representation learning is responsible for representing information as numerical vectors that can be processed by computers or further abstracted into higher-level feature vectors, multimodal representation learning refers to using the complementarity between multiple modalities to eliminate redundancy between modalities and thus learn a better feature representation [16]. The two main broad research directions are joint representation and cooperative representation. Joint representation maps multiple modal information together into a unified multimodal vector space, while collaborative representation is responsible for mapping each modality in a multimodal into its own representation space separately, and the mapped vectors satisfy certain correlation constraints among themselves.

Features obtained from multimodal representation learning are often used for information retrieval and classification/regression tasks. Modal transformation, also known as modal mapping, is responsible for transforming one type of modal information into another type of modal information. The most common current modal transformation approach is the encoding-decoding framework: using an encoder to represent the input as a semantic vector *C* and then using a decoder to transform the semantic vector *C* into a target output sequence. Common applications include machine translation and image description/video description. Machine translation is to translate the input from one natural language to another natural language on the fly; image description/video description is to form a textual description of a given image/video to express the content of the image/video. In a large number of optimization problems, there is more than just one optimal solution to the objective problem, and there may be multiple global and local optimal solutions, which is called multimodal optimization problem. A major feature of multimodal optimization compared to traditional optimization problems is that the solution algorithm is required to be able to provide all global and as many locally optimal solutions in the solution space in a single run.

In landscape design and green space maintenance scheduling systems, there are also many multimodal optimization problems to be solved. The MOA algorithm is a multimodal collaborative optimization algorithm, which is designed with multimodal group characteristics in mind and can be equated to the multicluster characteristics of the small habitat algorithm. In the algorithm, each queue node and its corresponding stack constitute a search group, as opposed to all search elements in the entire structure table, which represent the entire search tuple [17]. During the search process, each search group maintains its independence, and global information is exchanged only when the queue nodes are sorted. The ordering of the queue nodes only adjusts the allocation ratio of search resources, but each search group still keeps searching for an independent area. This design has two main purposes: to avoid the prematureness of the whole MOA algorithm during the search process because of falling into local optimal solutions and to support the use of multimodal optimization by using the characteristics of multivariate groups.

In contrast to the PSO algorithm for small habitats, the MOA algorithm has inherent multivariate group properties that allow it to be applied directly to multimodal optimization problems. During the operation of the MOA algorithm, each search group converges to a global or local peak. When the number of desired optimal solutions increases, the number of search groups can be increased by simply increasing the length of the MOA algorithm queue, bringing great simplicity to the use of the algorithm. Also, the algorithm avoids the increase in computational complexity due to the inherent multivariate group property compared to the small habitat algorithm. On the other hand, the MOA algorithm maintains the same mechanism of use in multimodal applications as in ordinary optimization, which avoids the addition of unfamiliar parameters, reduces learning costs, and eliminates the dependence on a priori experience. A large number of easy-to-score samples are detected in the previous branch network, and subsequent networks require fewer samples to be trained, which can significantly improve the computational efficiency of the network; each branch network can be trained to detect tree targets of different levels of difficulty, instead of being trained for the whole sample each time, resulting in the network not being able to learn the features of hard-to-score samples well. Thanks to the fact that the MOA algorithm stores the memory of the search process, and the algorithm has the feature of keeping the next generation of search elements not inferior to the current generation, the optimal solution will not be lost during the search process. At the end of the algorithm run search, all global and partial local optimal solutions can be taken out in the order of queue nodes from left to right.

Mask R-CNN is an instance segmentation framework inherited from Faster R-CNN, as shown in Figure 1, Mask R-CNN uses ResNet with a stronger characterization ability compared to Faster R-CNN instead of the VGG network and uses the updated FPN network instead of the RPN network to mine the feature-rich multiscale information. Mask R-CNN only adds a branch of Mask prediction to Faster R-CNN. Mask R-CNN uses the backbone network to extract features from the input image to get the feature map and then uses the FPN network to first make the feature map into a feature pyramid and then extract the ROI of the candidate regions from the different scales of the feature pyramid and finally needs to map the ROI of different scales back to the original image to get the final candidate regions. The mapping operation uses the ROI Align technique instead of the original ROI Pooling, whose main operation is to eliminate the rounding operation of ROI Pooling sampling so that the features obtained from each ROI can be better aligned with the ROI regions on the original map to get more accurate results for detection and localization [18]. Compared with traditional algorithms that rely on a priori knowledge, convolutional neural networks can automatically learn features from large amounts of data. Compared with shallow classifiers, convolutional neural networks build relatively complex network structures that combine feature extraction and classification training, mainly in terms of local perception and parameter sharing. The spatial connection of targets in images is more closely correlated among local pixels, while the correlation of distant pixels is weaker, so neurons can use local perception instead of global perception and finally combine all local information to get global information. In addition, each local region shares one convolutional kernel parameter, which simplifies the model training. The detection method based on the convolutional neural network (CNN) is more flexible and scalable and can be optimized for the characteristics of trees.

### 2.2. Application of Multimodal Intelligent Computing and Deep Neural Networks in the Construction of the Landscape Design and Greenery Maintenance Scheduling System

Landscape conservation and maintenance management and scheduling management are unified existences and cannot be separated. On the one hand, maintenance carries out every aspect of plant growth. Maintenance measures include planting, watering, fertilizing, spraying, pruning, mid-tillage, and others, mostly done directly by maintenance personnel or by manipulating machinery. On the other hand, the assigned maintenance tasks should achieve a reasonable distribution of time, the number of personnel, and workload. Managers should minimize the cost input of maintenance and management and reduce the waste of materials and labor [19]. When designing the landscape maintenance scheduling management system, the main purpose is to improve the corresponding efficiency. Therefore, the demand for the system's guarantee ability mainly requires the scalability, maintainability, and portability of the system application. Due to the current society, the ecological environment pressure is increasing continuously. Therefore, when designing this garden maintenance and scheduling management system, a long-term requirement needs to be designed to facilitate the system's functional services to be continuously increased in the subsequent process to meet the needs brought by the development of the garden. The main function structure of the system is shown in Figure 2.

The system can query different kinds of green plants in this base, which can be achieved by querying the name of green plants or related characteristics and also by combining queries. For green plants that have been delivered out, managers can delete them. Similarly, new plant species introduced to the base can be added and existing plants can be modified. Managers can make timely additions to maintenance records while automatically matching maintenance measures to green plants [20]. Maintenance records include records of all maintenance measures performed on plants, including pruning, mid-tillage, watering, planting, spraying, and fertilizing. We use a jump layer approach to reduce the upsampling step at the shallow level, use the results obtained here to fuse with the results obtained at the higher level, and finally perform one step of upsampling output and finally use deconvolution to complete the semantic feature manipulation of the whole landscape design. When browsing the basic plant information, you can see the plant family and the plant growth environment, and you can also choose to view the plant maintenance history, which is convenient for the administrator to record the maintenance history activities and better arrange future work tasks. The plant information function module can also realize task reminders for plants that have not been maintained for a long time according to the temperature and humidity in different seasons.

The structure of the progressive cascaded deep convolutional neural network based on this design is shown in Figure 3, in which the tree samples are divided into image batches and fed into each branch network in turn, and the last layer of each branch network is a Softmax layer to obtain a classification probability between 0 and 1 after the training of the branch [21]. At the same time, we set a set of positive and negative sample threshold intervals by grid search, that is, the previous branch network classification probability of the sample is within the positive and negative sample threshold interval, and the tree samples can be progressive to the next branch network to extract deeper tree features. The branch with a classification probability greater than the positive sample threshold can be labeled as easy positive sample filtering, and, similarly, the branch with a classification probability less than the negative sample threshold is labeled as easy negative sample filtering. For example, the first branch of the network has a lower classification probability for samples with a greater difference in color from the real trees and no obvious tree outline, so they are marked as the most easily classified negative samples by the first branch and given to the feature extraction module to reject the set of feature maps for these corresponding samples. Similarly, the positive samples that are most likely to be judged as trees by the network have a higher classification probability and are therefore marked as the most easily classified positive samples by the first branch and given to the corresponding feature extraction module. The remaining difficult samples are input to the second branch network to extract deeper features [22]. The second branch network is marked as the most easily scored negative samples for distracting backgrounds such as roads and buildings and is given to the set of extracted feature maps in the branch for rejection. The third branch can be dedicated to training the most difficult to score samples. We end up with a network structure where the dashed box is mainly the feature extraction module consisting of the convolutional and pooling layers in the three branches, and the dashed box below is mainly the branching module consisting of the other network layers in the three branches [23]. An additional advantage of this cascade network is that the feature maps can be partially shared. Since the main module and the branching modules are connected by the same cascade network, the feature maps obtained by extracting features can be fed to the branching modules to obtain classification probabilities for sample refinement and can also be advanced to the next branching network to extract deeper features without recalculating the original maps. Such a mechanism has two advantages: a large number of easy-to-classify samples are detected in the previous branch network, and the subsequent networks require fewer samples to be trained, which can significantly improve the computational efficiency of the network; each branch network can be trained to detect tree targets of different levels of difficulty, instead of being trained for the whole sample each time, resulting in the network not being able to learn the features of hard-to-classify samples well. Ultimately when three different networks work together, this can make the whole network more efficient.

Suppose that the number of image batches in each of our training processes is *γ*; our model has *X* branches, *p*(*x*, *y*) represents the *y* samples on the *x* branch in the image batch. Each branch network filters the samples corresponding to the difficulty of the image batches into two cases, as shown in the two following equations:

(1) $$\begin{array}{c} K_{\rho }\left(x,y\right)=\varphi \sum_{y\in \gamma }\sum_{x\in \chi }\left[p\left(x,y\right)\cdot \;\;\ln\;\;p\left(x,y\right)+Ax+Cy+\lambda \right], \end{array}$$

(2) $$\begin{array}{c} K_{\rho }\left(x,y\right)=\varphi \sum_{y\in \gamma }\sum_{x\in \chi }\left[\frac{p\left(x,y\right)}{\ln\;\;p\left(x,y\right)}-Ax-Cy\right]+\lambda . \end{array}$$

When the branch output probability is greater than the branch positive sample threshold is processed as a positive sample corresponding to the degree of refractoriness.

(3) $$\begin{array}{c} Rf\left(x\right)=\int \int g\left(t\right)\text{d}t\\ =\left(\frac{1+\gamma }{n}\right)\cdot \sum \left(x-1\right)f\left(t\right)+\lambda . \end{array}$$

When the branch output probability is less than the branch negative sample threshold is processed as a negative sample corresponding to the degree of refractoriness.

(4) $$\begin{array}{c} R^{m}f\left(x\right)=\int \int g\left(t\right)\text{d}t=\left(\frac{m+\gamma }{n}\right)\cdot \sum \left(x^{m}-t^{m-1}\right)f\left(t\right)+\lambda . \end{array}$$

Of course, accordingly, we will feed each branch filtered sample into the feature set in the feature extraction module, assuming *γ*_d_; then, we have

(5) $$\begin{array}{c} \gamma_{\text{d}}=\int \beta^{\text{Dirichlet}\left(\overset{⟶}{m}\right)}\cdot \eta^{r}\text{d}m. \end{array}$$

Our cascade network training process uses two stages of training: branch-level training and end-to-end training. The first stage is important because it can significantly accelerate the convergence speed of the later training in two ways: First, the later branch network will use the feature maps extracted by the previous network, so it can converge quickly. Second, for end-to-end training, branch-level training can initialize the parameters in the cascade network, so that only fine-tuning of the network parameters is needed for global training [24]. In branch-level training, we treat each branch network as a separate model for training. When the training of a branch network reaches a certain threshold of accuracy, we end the training by selecting the corresponding positive and negative sample thresholds to eliminate the easy samples, which will not be given to the next branch network. Correspondingly, the hard samples will go to the next network for feature extraction.

After getting the trained recursive cascaded convolutional neural network model, we need to collect the samples in the detected images with the help of the sliding window technique. The sliding window step size (the distance the sliding window moves in each step) will have a great impact on the final tree detection results. If the step size is too large, many trees will be missed and will not be detected. If the sliding step length is too small, the same tree target may be detected repeatedly [25]. The joint representation maps multiple modal information together into a unified multimodal vector space, while the cooperative representation is responsible for mapping each modality in the multimodal vector space into its respective representation space separately, and the mapped vectors satisfy certain correlation constraints among themselves. Moreover, the label prediction process will become very slow and inefficient due to the increase in the number of detections in the image. Through our experiments, it is more appropriate to set the step size to 2-pixel values in the detection process. For the samples obtained by the sliding window technique, a recursive cascade model is used for classification prediction and the trees are judged according to the classification probability output by the network.

### 2.3. Experimental Design

This experiment is to train and test the model based on a fully convolutional neural network for classifying feature elements in the landscape; firstly, the source of the training set of feature elements, preprocessing, and the implementation of the whole model is introduced, and the implementation form of the model built on Caffe framework and the training of the model is specified. Finally, the effect of semantic segmentation of the model is tested, and the accuracies of different upsampling structures are compared to determine the final model form for more accurate classification of feature elements in the landscape. The SIFT FLOW dataset was used for this experiment because the preparation time was too short, so there was no time to make the training set for training, so the SIFT FLOW dataset was used this time. The remaining 200 images will be used as the test set. The authors of the training set have classified the dataset into seven semantic categories, sky, mountain, plants, water, buildings, roads, and animals, according to the concept of urban design after the same kind of correction. The full depth neural network used in this paper mainly contains a convolutional layer (Convo-5), and a maximum pooling layer (Pool-7). Both use corrected linear units (ReLu) with sparse activation as the activation function. Convo-5 uses a stacked convolutional approach, with one or two identical convolutional layers stacked after each convolutional layer. To prevent overfitting and improve the robustness of the model, Conv6 and Conv7, which are followed by Dropout layers, are added so that a portion of the neuron outputs are zero and do not participate in network propagation to improve the generalization ability.

Because the deep learning full convolutional neural network is very complex, it will take more time in training, and the network level of a fully convolutional network is very deep, so the final result given by the model may remain near the optimal solution while conducting specific experiments, which may have an impact on the experimental results, and, on the other hand, it will make the convergence time of the whole model longer.

## 3. Results and Analysis

### 3.1. Analysis of Intelligent Distribution Results

After several iterations, the learning rate of the weight parameters was determined to be 10-10 and the weight decay coefficient was 0.005. The model training was conducted according to the given model training method, and the model second stage training method was not used for the comparison of the experiments. In the process of the model training method, 500 images of the training set were used as the pretraining dataset in the first stage, and then the model was trained in the second stage after that. The relationship between the loss and the number of iterations using the model training method and those without the model training method is shown in Figure 4.

The loss represents the value of the loss function, which is used to weigh the probability of which type of data is attributed to the test, and a lower loss function indicates that the network converges faster and faster. In Figure 4, we can see that the loss values of training with and without model stage 2 decreased rapidly from 300 to 500 iterations, but, after 500 iterations, the loss of the model training method reached 0.43 at 700 iterations, while it was only 0.47 without. Compared with shallow classifiers, convolutional neural networks build relatively complex network structures that combine feature extraction and classification training, mainly in terms of local perception and parameter sharing. The spatial connection of targets in images is more closely correlated among local pixels, while the correlation of distant pixels is weaker, so neurons can use local perception instead of global perception and finally combine all local information to get global information. The convergence rate of training with the model was significantly faster than that without model stage 2. The convergence speed of using model training is significantly faster than that of not using model two-stage training, which indicates that the convergence speed of using model training is flatter and flatter as the iteration proceeds, and finally both are in a more stable state, and the loss value after using model training is stable at about 0.41, while the loss value without using model training is stable at about 0.45, which indicates that the convergence speed of model training is flatter and flatter. The experimental results show that using model training can effectively accelerate the convergence speed of the training process of the semantic segmentation model of landscape images, and the data prove that the method is practical and feasible.

As shown in Figure 5, here are the results of semantic segmentation of garden design features by each of the three upsampling structures, with the top of the figure indicating the features corresponding to different semantic categories. It is obvious from the figure that FCN-8S is more prominent than the other two upsampling structures. The drawback of the final output image of FCN-32S in the figure is that the edge segmentation is not very good and lacks some detailed information, and the detail processing part is very poorly done. For this reason, this paper uses the method of jumping layers here, reducing the upsampling step in the shallow layer, using the results obtained here to fuse with the results obtained in the higher layer, and finally performing one step of upsampling output and finally using deconvolution to complete the semantic feature operation for the whole garden design. From the figure, we can see that FCN-16S has great improvement over FCN-32S, and FCN-8S is more excellent than FCN-16S in terms of detail processing, so the best upsampling structure FCN-8s is selected for this thesis in terms of feature semantic classification in landscape design.

## 4. Instance Verification

In landscape design, there is a mutually constraining relationship between project duration, cost, quality, safety, and environmental protection level, of which the cost is most affected by the duration, and the shortening of the duration requires the investment of more mechanical and labor resources. This will lead to an increase in costs, but in the long run, it will lead to an increase in indirect costs such as overhead, which will also lead to an increase in costs. And with the improvement of the security level, the cost that needs to be paid is also getting higher and higher. When the duration is sufficient, the quality level and environmental protection level of the project are also guaranteed. The project decision-maker can choose the best option based on the project's specific requirements for the duration, cost, quality, safety, and environmental protection and allocate resources for the implementation of each process. To more intuitively represent the decision options given by these six optimization schemes and more visually show the distribution of the Pareto solution obtained by solving the model with the multiobjective elite inverse golden sine whale algorithm, the three-dimensional spatial diagram of “duration-cost-quality, safety, and environmental protection water average” is shown in Figure 6.

As can be seen from Figure 7, compared with the basic project requirements, the optimization solutions given by both algorithms have a more positive impact on the achievement of each project goal to a certain extent, and the optimization effect of the improved algorithm proposed in this paper is more obvious compared with the basic whale algorithm. Among them, Option 1 has the best optimization in the schedule goal, with an optimization degree of 25.71%; Option 3 has the best optimization effect on the cost, with an optimization degree of 21.28%; Option 4 has the best optimization effect in the safety goal, with the optimization degree of 24.93%; Options 5 and 6 have the best optimization degree of 16.4% in the quality; in addition, Option 6 has the best optimization effect in the environment. It is worth noting that Option 6 performs better in quality, safety, and environmental objectives.

When the number of solutions stored in external green plants reaches the upper limit of green plant storage, the crowding distance value between solutions is calculated, and the solutions with smaller distance values in the green plant are deleted according to the ranking of the crowding distance. This method has two shortcomings. On the one hand, deleting multiple solutions with small distance values at one time will lead to the change of the crowding distance values of the remaining solutions to have a greater impact on the green plants, and deleting multiple solutions with small distance values at one time will also lead to the overall truncation of a region where the solutions are more concentrated, thus affecting the distribution of the solution population and leading to an uneven distribution of the solution set. On the other hand, as shown in Figure 8, if the crowded distance mechanism is used to maintain the green plants, both *B* and *C* will get a large crowded distance value and thus be preserved as sparse individuals, but, in fact, *B* and *C* are very close to each other in the target space and belong to the dense area, so the crowded distance mechanism can hardly reflect the real distribution of the solution set.

It is obvious from the value index of each index in Figure 9 that the value index of road plaza paving, lawn ground cover planting, and tree planting is slightly smaller than that which indicates that the cost of forming this function is slightly higher and some costs need to be reduced appropriately. The value index of garden buildings, garden terrain, and shrub planting is slightly greater than that indicating that their corresponding allocated costs are less, or their functions are slightly richer, and the capital investment of garden service buildings should be appropriately increased within a reasonable range to meet the functional needs of people to a greater extent.

With the help of modern management technologies such as multimodal intelligent computing and deep neural networks, a sufficient number of diverse options for quality landscape design and greenery maintenance can be generated to meet the requirements of each goal, providing decision support for enterprises, which can then choose the right one among the options according to their own needs.

## 5. Conclusion

In this paper, from a practical problem, we introduce multimodal intelligent computing and deep neural network algorithm for the segment of urban indoor greening and design and implement a three-dimensional green plant maintenance system for indoor greening. It realizes the main functions of three-dimensional planting and maintenance, real-time plant information monitoring, remote control, and so forth. Users can observe the growth condition of green plants in real time through the network and maintain the plants remotely, which provides a new idea for further promotion of urban indoor greening. Through the practice of digital landscape design methods in landscape design projects, the advantages of digital landscape design for landscape gardening can be seen; designers select the content of landscape target analysis according to the type of site and then establish specific parametric models with the help of digital tools, transform two-dimensional information into three-dimensional information with data analysis and parametric modeling, construct an accurate relationship through data, and convert complex spatial information into the understandable parametric model; fully grasp the advantages and disadvantages of the site in the scheme design stage, which greatly improves the scientific and logical landscape design.

At present, the research content of the wisdom garden mainly focuses on the development and application of the wisdom management system and also includes the initial application of intelligent systems such as intelligent light system, intelligent water system, and intelligent plant watering system. The development of the digitalization of smart gardens also requires the joint efforts of peers and scholars in this profession. Garden design requires the organic combination of smart technology and designers, participants, and professionals in other fields. This is a new way of garden design and a major trend in the future development of gardens. For the research content of the digital design of the smart garden, in addition to the further deepening of the digital design method, all aspects of the future application of digital technology also need to be carried out simultaneously.

## Figures and Tables

**Figure 1:** Mask R-CNN segmentation framework diagram.

**Figure 2:** System main function framework diagram.

**Figure 3:** Recursive cascaded deep convolutional neural network structure.

**Figure 4:** Relationship between loss values and number of iterations.

**Figure 5:** Semantic segmentation results of landscape design features.

**Figure 6:** “Duration-cost-quality, safety, environmental protection water average” three-dimensional chart.

**Figure 7:** Comparison of the optimization effect of landscape design and construction plan.

**Figure 8:** Congestion distance mechanism.

**Figure 9:** Value index of each indicator.

## Data Availability

The data used to support the findings of this study are available from the corresponding author upon request.
